The article "Structural equation modeling to estimate treatment adherence based on the light triad of personality and sense of coherence in patients with type-2 diabetes: examining the mediating role of psychological well-being" was retracted in 2024. Reasons: original data or images not available; unreliable data; concerns about the data.

# Structural equation modeling to estimate treatment adherence based on the light triad of personality and sense of coherence in patients with type-2 diabetes: examining the mediating role of psychological well-being

**DOI:** 10.3389/fpsyg.2023.1285808

**Published:** 2023-11-27

**Authors:** Seyedeh Maryam Mousavi, Seyedeh Masoumeh Bagheri, Nasrin Jalali Heris, Parisa Matbouraftar, Mozhdeh Azarian, Mohammadreza Kordbagheri

**Affiliations:** ^1^Department of Nursing and Midwifery, Rasht Branch, Islamic Azad University, Rasht, Iran; ^2^Lahijan Branch, Islamic Azad University, Lahijan, Iran; ^3^Rasht Branch, Islamic Azad University, Rasht, Iran; ^4^Department of Statistics, Faculty of Mathematical Sciences, Shahid Beheshti University, Tehran, Iran

**Keywords:** personality traits, diabetes mellitus, psychological well-being, SEM, light triads

## Abstract

**Background:**

The current study investigated the relationship between the light triad of personality and self-coherence with treatment adherence in patients with Type 2 Diabetes Mellitus (T2DM) using Structural Equation Modeling (SEM). Psychological well-being was considered a mediator variable in this SEM assessment.

**Method:**

A cross-sectional study by convenience sampling was conducted, and 368 patients with T2DM were recruited from 10 private practice and general hospitals from May to November 2021 in Gilan province, Iran. The Reef’s Psychological Well-being Questionnaire, the Light Triad Rating Scale, and Antonovsky’s Sense of Coherence Scale were used for data collection. Structural equation modeling was used to examine the model fitness and identify direct/indirect relationships among variables. Data were analyzed by the SPSS (Version 26) and AMOS software (Version 24).

**Results:**

The average score of light triads, sense of coherence, psychological well-being, and treatment adherence were 70.36 ± 25.55, 108.25 ± 37.68, 57.03 ± 23.84, and 106.81 ± 39.61, respectively. Model fit statistics suggest that the measurement model fits the data well: χ2 (146, *N* = 368) = 314.011 (*p* < 0.001). The SEM results showed that the light triad of personality (β = 0.12) and self-coherence (β = 0.14) were positively associated with treatment adherence. Anxiety, the light triad of personality (β = 0.12), and self-coherence (β = 0.14) affect treatment adherence indirectly through psychological well-being.

**Conclusion:**

The analysis of the SEM revealed that the suggested model had a suitable goodness of fit. So, using self-coherence and psychological well-being structures in designing interventional programs is recommended to optimize treatment adherence in patients with T2DM.

## 1 Introduction

The World Health Organization states that over 422 million people worldwide have been diagnosed with diabetes (World Health Organization, 2021). Approximately 90% of all patients diagnosed with diabetes are classified as having Type 2 diabetes mellitus (T2DM) (Kumar and Mohammadnezhad, 2022).

Various studies indicate that diabetes health management encompasses activities such as carbohydrate counting, daily monitoring of insulin dosage, scheduling daily exercise routines, and engaging in psycho-educational sessions (Winkley et al., 2020; Davoudi et al., 2021). This set of activities is called treatment adherence (Hamine et al., 2015). Treatment adherence is the degree to which a patient’s behaviors align with practitioner recommendations, including adhering to dietary guidelines, medication management, and implementing recommended environmental changes (Alqarni et al., 2018). Recently, a meta-analysis showed that diabetes distress, cognitive impairment, anxiety, poor communication with practitioners, older age, concerns about medicines, and stress highly correlated to treatment adherence in patients with T2DM (Świątoniowska-Lonc et al., 2021). Indeed, improving treatment adherence could be a suitable target for enhancing the quality of life for patients with T2DM.

Recently, personality has gained recognition as a significant variable for predicting treatment adherence. For example, one study demonstrated a notable negative correlation between neuroticism personality traits and treatment adherence in patients with T2DM (Bayat Asghari et al., 2015). Furthermore, emotional stability and consistency were predictors of higher treatment adherence levels in these patients (Novak et al., 2017). People with different personality characteristics may approach treatment and medication adherence differently (Cheli et al., 2022). So, understanding these differences can help healthcare providers better tailor treatment plans to suit individual needs (Bruce et al., 2010). Also, considering personality as a variable in predicting treatment adherence allows healthcare providers to take a more holistic and personalized approach to patient care (Bagby et al., 2016).

Within the realm of personality traits, the dark triad of personality has garnered attention in the context of adverse health outcomes (Gogola et al., 2021). The dark triad personality encompasses narcissism, machiavellianism, and psychopathy (Kowalski et al., 2021). In treatment adherence, numerous studies have examined potential associations between the dark triad of personality and compliance with health-related policies and guidelines (Carvalho and Machado, 2020; Chávez-Ventura et al., 2022; Morales Vives et al., 2023). For instance, one study identified that narcissism, a constituent of the dark triad of personality, plays a substantial negative role in adherence to the Coronavirus Disease of 2019 (COVID-19) health-related behaviors (Vaal et al., 2022).

A set of traits opposite to the dark triad of personality includes light personality traits. The light personality traits typically refer to positive qualities, attitudes, and behaviors associated with empathy, compassion, altruism, and other virtues that promote well-being and positive interactions with others (Alipour Gourand et al., 2022). These traits contrast with the Dark Triad traits, which encompass narcissism, machiavellianism, and psychopathy, known for their more negative and self-centered characteristics (Mejía-Suazo et al., 2021; Grigoropoulos, 2023). Light personality traits emphasize qualities that contribute to positive social interactions and relationships. Light personality traits can significantly influence adherence to health-related behaviors for several compelling reasons. Individuals with these traits often exhibit enhanced motivation to prioritize their health, driven not only by self-concern but also a genuine care for the well-being of others (Baldacchino, 2023). Their ability to form and seek social support is another crucial factor, as a strong support system can provide encouragement, reminders, and accountability, reinforcing their commitment to adhering to recommended health guidelines (Mejía-Suazo et al., 2021). Besides, there is limited knowledge regarding the influence of light personality traits on adherence to health-related behaviors and policies. For instance, self-reported adherence was found to positively correlate with the light core of personality in COVID-19 health-related behaviors (Grežo and Adamus, 2022). To the best of our knowledge, there is no study about the role of light triad personality traits in adherence to treatment in patients with diabetes. Nevertheless, determining the role of the light triad core in treatment adherence dimensions can play an essential role in developing new behavioral treatments in patients with diabetes.

Another possible structure that plays an essential role in treatment adherence is the “Sense of Coherence (SOC).” SOC includes manageability, comprehensibility, and meaningfulness (Pallant and Lae, 2002). Manageability refers to the perception of the available internal resources to cope with (or respond) to external demands (Pallant and Lae, 2002). Understanding what happens when a person is exposed to pleasurable or stressful stimulation is called comprehension. Finally, meaningfulness (the core of SOC) is the motivation that inspires people to find the resources they need to cope with a specific situation (Arvidsdotter et al., 2016). Previous results showed higher levels of SOC associated with better treatment adherence. For example, one study showed that SOC could predict treatment adherence, disease activity, and function in patients with systemic lupus erythematosus (Duvdevany et al., 2011). In the context of diabetes, one study showed positive correlations among treatment adherence, SOC, and illness acceptance in these patients (Alyami et al., 2019). However, a scant empirical inquiry has been conducted on the correlation between treatment adherence and SOC among patients with T2DM. So, it is necessary to evaluate this association in the same population. On the other hand, the results of various studies have shown that psychological well-being can mediate the relationship between SOC, personality, and treatment adherence (Bajwa and Shoukat, 2019; Silva et al., 2021; Rana et al., 2022).

### 1.1 Research hypothesis

In summary, light triad and SOC are associated with better adherence to treatment. In addition, these structures are associated with psychological well-being, and psychological well-being can play an essential role as a mediator in these associations. So, we proposed a treatment adherence model (see Figure 1) in patients with T2DM. Psychological well-being mediates the relationship between the light triad of personality and a SOC with treatment adherence in patients with T2DM.

**Figure 1:** Proposed model.

*Hypothesis 1:* Psychological Well-Being mediates the association between the light triad of personality and treatment adherence.

*Hypothesis 2:* Psychological Well-Being mediates the association between the sense of coherence and treatment adherence.

## 2 Method

### 2.1 Study design

A cross-sectional design was used in the present study to estimate treatment adherence based on the light triad of personality traits, SOC, and psychological well-being in patients with T2DM. This study was conducted from May to November 2021 in Gilan, Iran.

### 2.2 Participants and study criteria

The participants of this study included 368 patients with T2DM (between 40 and 70 years) who met the T2DM criteria, according to the American Diabetes Association. We focused our analysis on a specific age range to mitigate the potential influence of age-related effects on patient’s complaints and symptoms.

The sample consisted of patients with T2DM who were voluntarily selected and met the eligibility criteria for the current study. Three centers within Gilan Province, Iran, were selected from the region’s general hospitals. Additionally, we sent advertising letters to private medical practices, inviting patients to participate in the current study. To facilitate communication and address potential participants’ inquiries, we provided a contact number (belonging to the corresponding author). Ultimately, invitations were extended to 500 patients, of which 368 met the inclusion criteria and responded to our call.

Inclusion criteria were as follows: (a) receiving a T2DM diagnosis by a physician; (b) being between 40 to 70 years old; (c) having reading and writing literacy; (d) willingness to study participation; (e) not having Alzheimer’s disease or dementia. Three hundred sixty-eight patients [females (35.96%)] with a mean age of 56.01 ± 8.84 have participated in the present study. The HbA1c range was between 6.10 and 15. Table 1 presents the sociodemographic variables of the patients.

**Table 1:** Basic description of the sociodemographic variables in the study participants.

Variable		Mean ± SD / *N* (%)
Age		56.01 ± 8.84
Gender	Male	232 (63.04%)
	Female	136 (35.96%)
HbA1c		8.73 ± 1.94
Educational level	Primary School or below	138 (37.5%)
	High school	186 (50.5%)
	Bachelor’s or higher	44 (12%)
Marital status	Single	16 (4.3%)
	Married	270 (73.4%)
	Divorced	12 (3.3%)
	widow	70 (19%)
Job-status	Full time	111 (30.2%)
	House-keeping/ Unemployed	182 (49.5%)
	Retired	63 (17.1%)
	Part-time	12 (3.2%)
Disease duration (years)	>5	103 (27%)
	6–10	158 (42.9%)
	10≥	107 (29.1%)

### 2.3 Measures

- *Sociodemographic and clinical variables*: We evaluated age, gender, Hemoglobin A1C, marital status, disease duration, education level, and job status in the present study. Age and disease duration are considered continuous variables (years). Options for education levels included “primary school or below,” “high school,” and “bachelor’s or higher.” Also, we categorized marital status as “single,” “married,” “divorced,” and “widow.” HbA1c was recorded from the patient’s documents. In order to develop a demographic and clinical checklist, we used previous studies’ guidelines in the context of diabetes (Davoudi et al., 2021; Rajaeiramsheh et al., 2021).
- *Light Triad Personality*: The original version of light triad personality traits was developed by Johnson as their master of science in psychology at the University of Western Ontario. For more information about this scale, its items, and the original version’s psychometric properties, please refer to Johnson (2018). This scale has three subscales include: altruism, compassion, and empathy. The light triad of personality scale scoring method is a five-point Likert scale (from totally disagree = one to agree = five totally). In the current study, the Persian version of this scale presented suitable psychometric properties (internal consistency = 0.8, test–retest reliability = 0.91). In the current study, Cronbach’s alpha value was estimated at 0.876.
- *Treatment adherence*: A 40-item scale for evaluating treatment adherence levels among patients with chronic diseases has recently been developed. This scale developed into Persian (the language of patients who participated in the current study) and exhibited favorable psychometric properties when applied to individuals with chronic diseases. This scale has seven subscales, including due diligence in the treatment process, willingness to engage in treatment, adaptability, integration of treatment into daily life, adherence to treatments, commitment to treatment, and hesitation to seek treatment. [For access to the items and their psychometric properties, please see (Seyed Fatemi et al., 2018)].
- *Sense of Coherence*: Antonovsky (1987) created a survey to assess the perception of coherence. The initial version, known as the Orientation to Life Questionnaire, comprises 29 items about “understanding,” “ability to handle situations,” and “sense of significance.” For more information about this scale, its items, and the original version’s psychometric properties, please refer to Antonovsky and Sagy (1986). Respondents provide their answers on a semantic scale ranging from 1 to 7 points. The Persian version of this scale showed suitable psychometric properties (Alipour and Sharif, 2012). In the current study, Cronbach’s alpha value was 0.832.
- *Psychological well-being*: The evaluation of well-being is conducted through an adapted 18-item variant of Ryff’s scales of psychological well-being. This scale incorporates three inquiries for each of the six facets of well-being, namely self-acceptance, autonomy, environmental mastery, purpose in life, positive relations with others, and personal growth [for more information, items, and psychometric properties of the original version, please see (Wilson et al., 2013)]. This questionnaire score ranges from one (strongly disagree) to six (strongly agree). Higher scores indicate higher levels of PWB. According to Khanjani et al., the internal consistency of PBQ-18 was estimated at 0.71, which means this scale is suitable for use in the Iranian context (Jahan and Nematolahi, 2021). In the current study, Cronbach’s alpha value was 0.91.

### 2.4 Analytic plan

We used a suggested criterion for sample size determination (5–20 respondents for every parameter) (Bentler and Chou, 1987). This study had 39 free parameters; the estimated sample size was 368 patients.

First, descriptive statistics were estimated to include mean, standard deviation, kurtosis, and skewness. All research variables’ skewness and kurtosis values were from −3 to +3, confirming normal distribution. Pearson’s bivariate and Tetrachoric correlations were subsequently used to estimate the associations among the variables. These analyses were conducted using the SPSS software (Desktop version 26). Second, the main aim of the present study was to investigate the relationship between variables based on structural equation modeling in AMOS 24 (Byrne, 2016). In addition, the maximum likelihood method has been used to estimate the parameters. In statistics, maximum likelihood estimation (Kessler et al., 2005) is a method of estimating the parameters of an assumed probability distribution given some observed data. This is achieved by maximizing a likelihood function so that the observed data is most probable under the assumed statistical model. Data on 368 participants were initially examined for outliers and normality. Univariate outliers (z scores greater than 3.29 and less than −3.29) were excluded from analyses (Kline, 2023). Multivariate outliers were non-problematic (D2 values were not distinctively apart (Byrne, 2016), which resulted in a sample of 368 participants. Multivariate normality was confirmed (multivariate kurtosis critical ratio was less than 5.00). Bootstrap analyses were conducted using the recommended bias-corrected (BC) confidence intervals (Hugtenburg et al., 2013) and 5,000 bootstrap samples (Bollen and Stine, 1992). To evaluate the model fit, we used the comparative fit index (CFI) > 0.9, Incremental Fit Index (IFI) > 0.9, Goodness of Fit Index (GFI) > 0.9, Parsimonious Comparative Fit Index (PCFI) > 0.5, Parsimonious Normed Fit Index (PNFI) > 0.5, the standardized root means square residual (SRMR) < 0.08, and the root mean square error of approximation (RMSEA) < 0.08 (Kline, 2023). Furthermore, we calculated the coefficient of determination (*R^2^*) to estimate the proportion of the variance in the dependent variables explained by the independent variables (Marsh and Scalas, 2018).

## 3 Results

At first, the variable measurement part of the proposed model was evaluated based on confirmatory factor analysis. In the following, the descriptive indices and correlation between the variables were investigated, and finally, the structural model of the research was evaluated. The results of the direct and indirect effects of the proposed model were reported.

### 3.1 Confirmatory analysis

We used Confirmatory Factorial Analysis (CFA) estimation to evaluate scale appropriateness in our study. Acceptable fit indexes were obtained for Light Triad [χ2/df = 2.96; CFI = 0.90; IFI = 0.91; GFI = 0.92; PCFI = 0.54; PNFI = 0.54; RMSEA = 0.07 (0.06–0.09); SRMR = 0.03], SOC [χ2/df = 2.35; CFI = 0.96; IFI = 0.97; GFI = 0.98; PCFI = 0.62; PNFI = 0.63; RMSEA = 0.06 (0.05–0.08); SRMR = 0.02], psychological well-being [χ2/df = 2.12; CFI = 0.97; IFI = 0.97; GFI = 0.98; PCFI = 0.63; PNFI = 0.64; RMSEA = 0.05 (0.04–0.07); SRMR = 0.02] and treatment adherence [χ2/df = 2.88; CFI = 0.93; IFI = 0.93; GFI = 0.94; PCFI = 0.59; PNFI = 0.58; RMSEA = 0.07 (0.06–0.08); SRMR = 0.06]. In addition, the factor loading of the items of each component was higher than 0.4 (Sarstedt et al., 2021). These results indicated that the scales used in this study have acceptable validity and reliability.

### 3.2 Correlation among variables

Table 2 shows a significant relationship between the light triad of personality and SOC with psychological well-being and treatment adherence. Also, there was a significant relationship between psychological well-being and treatment adherence. The results of the Tetrachoric Correlation test showed no significant difference between the levels of adherence to treatment regarding education level, employment status, gender, marital status, and duration of illness (*p* > 0.05). Also, there was no significant correlation between age and hba1c with treatment adherence scores (*p* > 0.05).

**Table 2:** Descriptive statistics and correlation among main variables.

	1	2	3	4
1. Light triad	1			
2. Sense of coherence	0.57**	1		
3. Psychological well-being	0.42**	0.56**	1	
4. Treatment adherence	0.57**	0.34**	0.34**	1
M	70.36	108.25	57.03	106.81
SD	25.55	37.68	23.84	39.61
skewness	−0.05	−0.26	0.04	0.01
kurtosis	−1.15	−1.20	−1.29	−1.30

**p < 0.001. *N* = 350. M, Mean; SD, standard deviation.

### 3.3 Tests of hypothesized model and mediation analyses

In line with the current research’s main goal, Anderson and Gerbing’s two-step approach was used (Anderson and Gerbing, 1992). First, the fitness of the proposed model was evaluated based on Confirmatory Factor Analysis (CFA). Second, the proposed model was tested based on structural equation modeling. Model fit statistics suggest that the measurement model fits the data well: χ2 (146, N = 368) = 314.011, *p* < 0.001; CFI = 0.95; SRMR = 0.05; RMSEA = 0.05, 90% CI [0.04, 0.07]; PNFI = 0.58; PCFI = 0.59; IFI = 0.96 and GFI = 0.90. All factor loadings were significant at *p* < 0.001. The hypothesized model was also acceptable for the data χ2 (146, N = 368) = 314.011, *p* < 0.001; CFI = 0.95; SRMR = 0.05; RMSEA = 0.05, 90% CI [0.04, 0.07]; PNFI = 0.57; PCFI = 0.58; IFI = 0.97 and GFI = 0.91. Figure 2 presents the three latent variables’ key estimated structural model paths and factor loadings.

**Figure 2:** The model with standardized estimates.

### 3.4 Direct paths

The results showed that the light triad of personality and SOC had a positive and significant effect on psychological well-being and treatment adherence (see Table 3) (*p* < 0.001). Therefore, with the light triad of personality and SOC increase, psychological well-being and Treatment adherence. Also, the results showed that psychological well-being has a positive and significant effect on Treatment adherence (β = 0.34; *p* < 0.001). Therefore, with the increase in psychological well-being, the levels of treatment adherence will increase. The model tested (Table 3) explains 50% (*R*^2^ = 0.50) of the variance in treatment adherence and 32% of the variance in psychological well-being (*R*^2^ = 0.32) (Kline, 2023).

**Table 3:** Direct effects among variables.

Path estimate	Path coefficient	*SE*	*CR*	*p*
Direct effect				
Light triad of personality --- > Psychological well-being	0.35	0.01	5.12	<0.001
Light Triad of Personality --- > Treatment adherence	0.57	0.09	11.31	<0.001
Sense of coherence --- > Psychological well-being	0.40	0.01	6.77	<0.001
Sense of coherence --- > Treatment adherence	0.23	0.03	4.02	<0.001
Psychological Well-Being --- > Treatment adherence	0.34	0.01	5.01	<0.001
Squared multiple correlation (*R*^2^):				
Psychological well-being	0.32			
Treatment adherence	0.50			

### 3.5 Indirect paths

The determination of mediation in the model was based on examining the significance of the indirect effects of the bootstrap procedure. Two indirect relationships were significant (Table 4). Table 4 shows that psychological well-being mediates the relationship between the light triad of personality (β = 0.12; *p* < 0.001) and SOC (β = 0.14; *p* < 0.001) with treatment adherence. In other words, the relationship between the light triad of personality and SOC with treatment adherence has increased with the inclusion of the psychological well-being variable.

**Table 4:** Indirect effects among variables.

Path estimate	Path indirect	SE.	95% BC CI	
			Lower	Upper
Indirect effect				
Light triad--- > Psychological well-being--- > Treatment adherence	0.12**	0.01	0.05	0.18
SOC --- > Psychological well-being--- > Treatment adherence	0.14**	0.02	0.07	0.21

BC CI, bias-corrected confidence intervals. Bold: Significant. **p < 0.05. **p < 0.01.

## 4 Discussion

We aimed to evaluate the associations among light triad traits, SOC, and treatment adherence in patients with T2DM. Additionally, we examined the potential mediating effect of psychological well-being on the relationship between light triad traits and SOC with treatment adherence. This study is significant as there is a lack of literature on this topic concerning T2DM patients. The findings of the predict treatment adherence in patients with T2DM. We tried to provide some details about the findings in the following lines.

First, the results revealed significant direct effects of the light triad on treatment adherence. We found that light personality traits could influence treatment adherence levels. This finding aligns with previous studies. For instance, one study demonstrated a positive relationship between adherence to COVID-19 containment measures and the light triad of personality traits, consistent with our study’s results (Grežo and Adamus, 2022). This procedure can be attributed to several factors. Firstly, patients’ heightened empathy (as a subscale of the light triad of personality) fosters a genuine concern for their well-being as well as the well-being of others, motivating them to prioritize health-related recommendations. Secondly, patients’ ability to form strong social support networks is crucial (Jones and Huggins, 2014; Cieślik et al., 2023). These networks provide encouragement, reminders, and accountability, reinforcing their dedication to adhering to recommended health guidelines. Lastly, their altruistic tendencies lead them to prioritize their health for personal reasons, set positive examples, and ensure they can continue caring for loved ones. These traits collectively contribute to their greater adherence to treatment regimens (Ramos-Vera et al., 2023).

Secondly, we discovered that psychological well-being could mediate the association between light triad personality traits and treatment adherence levels. This study marks the first attempt to calculate this pathway, and as such, there were no similar studies in the existing research literature. However, previous studies have indicated that compassion, considered a light personality trait, is positively associated with psychological well-being (Jones and Huggins, 2014). Additionally, these studies have shown that psychological well-being is significantly linked to treatment adherence (Bąk-Sosnowska et al., 2022).

These findings bear some resemblance to our own. Our research revealed that psychological well-being can mediate the relationship between light triad personality traits and treatment adherence levels for several reasons. Firstly, individuals with higher levels of light triad traits like empathy, compassion, and altruism tend to experience greater psychological well-being (Jones and Huggins, 2014). These positive personality traits reduce stress, anxiety, and depression, creating a more conducive mental environment for adhering to treatment regimens (Carvalho and Machado, 2020). Secondly, psychological well-being enhances an individual’s overall sense of self-efficacy and control over their health, fostering the belief that they can successfully follow treatment recommendations. This increased self-confidence translates into improved adherence behavior. Lastly, psychological well-being often leads to a more positive outlook on life, making individuals more inclined to engage in health-promoting behaviors, including adherence to treatment plans. Therefore, psychological well-being mediates by positively influencing the light triad traits and treatment adherence levels (Carvalho and Machado, 2020; Cieślik et al., 2023).

Third, we found that SOC has a significant correlation with treatment adherence. This result is the line of previous studies. In one study, researchers found that SOC could significantly affect self-report treatment adherence levels in the context of COVID-19 Pandemic restrictions among infected patients (Novak et al., 2022). In another study, authors found that SOC could predict medication adherence, which was in line with our findings (Tyer-Viola et al., 2014).

The significant correlation between SOC and treatment adherence can be attributed to several underlying factors. First, individuals with a higher SOC tend to possess a stronger internal locus of control and a greater ability to make sense of and cope with various life stressors, including health-related challenges (da-Silva-Domingues et al., 2022; Jeserich et al., 2023). This heightened psychological resilience translates into a more positive and proactive approach to managing their health, making them more likely to adhere to treatment plans. A strong SOC is often associated with a heightened sense of purpose and meaning in life. Individuals with a clear sense of purpose may view adhering to treatment regimens as a means of preserving their overall well-being and achieving their life goals. This intrinsic motivation fosters a greater commitment to treatment adherence (Poursalehi et al., 2021; Langeland et al., 2022).

Fourth, we found that psychological well-being could mediate the association between SOC and treatment adherence. Finally, we found that SOC and light triad of personality had significant and positive associations. These results are consistent with previous studies. For instance, one study found a significant association between SOC and psychological well-being (Nilsson et al., 2010). Furthermore, we discussed the association between psychological well-being and treatment adherence in the preceding sentences. We did not find a similar conducted study on the association between SOC and the light triad, but it could be justified by previous literature.

The association between SOC and the light triad of personality traits can be elucidated through several interconnected pathways (Langeland et al., 2022). Individuals with a higher SOC tend to experience greater psychological well-being, marked by reduced stress, anxiety, and depression, which may nurture the development of light triad traits like empathy, compassion, and altruism (Novak et al., 2022). Moreover, a strong SOC often fosters a positive worldview, leading to a heightened inclination to exhibit these prosocial traits and engage in altruistic actions (Poursalehi et al., 2021). Furthermore, SOC equips individuals with effective coping mechanisms, enabling them to navigate life’s challenges while preserving their empathetic and compassionate tendencies. This adaptability and resilience, coupled with a sense of purpose often associated with a robust SOC, contribute to the sustained expression of light triad traits, illustrating the intricate relationship between SOC and these virtuous personality characteristics (Pallant and Lae, 2002).

### 4.1 Limitations and future directions

Besides promising results, the present study faced some limitations. First, because of the cross-sectional nature of this study, we could not infer causality among variables. So, future studies should use experimental designs to analyze the causal mechanisms underlying the interactions among variables in depth. Second, the results are extracted from the self-report of the patients with T2DM, and the conclusions are based on a representative sample of Northern Iran, which limits the generalization of the results to other populations. Finally, the self-report method performed by patients is loaded with tendencies that link the responses to remembered experiences; thus, future studies should ensure that patients report on the study variables after some program that will increase the accuracy of the reports.

## 5 Conclusion

The results of the present study showed that psychological well-being plays a mediating role in the relationship between the light triad of personality and SOC with treatment adherence. According to previous literature, the light triad of personality traits and SOC are associated with positive psychological constructs such as hope, gratitude, self-regulation, mature defense mechanisms, and emotional stability. These positive psychology components can lead to more health-promoting behaviors and increase psychological well-being. These results are partially consistent with previous research. For example, Chilver et al. showed that personality components (lower levels of neuroticism and higher levels of conscientiousness) and cognitive reappraisal could predict better psychological well-being (Chilver et al., 2023). Although these components were not directly examined in the current research, most components related to the light triad of personality traits and SOC have a structure similar to low neuroticism and high conscientiousness.

On the other hand, patients with higher psychological well-being usually show higher spontaneity and a healthier lifestyle (Bożek et al., 2020). As a result, in a healthy cycle of self-reinforcement, the probability of their adherence to treatment increases, and this issue was shown in the present study among patients with diabetes. Based on this, clinicians must pay attention to the role of the light triad of the personality of personality, SOC, and psychological well-being in treating patients with T2DM. Developing interventions to improve these traits is also suggested, if possible, and patients at risk should be identified early.

## Data availability statement

The original contributions presented in the study are included in the article/Supplementary material, further inquiries can be directed to the corresponding author.

## Ethics statement

Ethical review and approval was not required for the study on human participants in accordance with the local legislation and institutional requirements. The studies were conducted in accordance with the local legislation and institutional requirements. The participants provided their written informed consent to participate in this study.

## Author contributions

SM: Writing – original draft. SB: Writing – review & editing. NJ: Writing – review & editing. PM: Writing – review & editing. MA: Writing – review & editing. MK: Data curation, Methodology, Software, Validation, Writing – original draft.
